This article has been retracted.

# Nurses’ Attitudes Toward Psychiatric Help for Depression: The Serial Mediation Effect of Self-Stigma and Depression on Public Stigma and Attitudes Toward Psychiatric Help

**DOI:** 10.3390/ijerph17145073

**Published:** 2020-07-14

**Authors:** Eunmi Lee, Yoo Mi Jeong, Su Jeong Yi

**Affiliations:** 1 Department of Nursing, Research Institute for Basic Science, Hoseo University, Asan-si 31499, Korea; sweetbear2@hanmail.net; 2 College of Nursing, Dankook University, Cheonan-si 31116, Korea; 12181056@dankook.ac.kr

**Keywords:** depression, seeking help, stigma, nurse

## Abstract

This study aimed to examine the mediating effects of self-stigma and depression on the public stigma and nurses’ attitudes toward psychiatric help. A cross-sectional study with 184 nurses at one general hospital in South Korea was conducted employing a self-administered survey, using the Attitudes toward Seeking Psychological Help Scale, the Beck Depression Inventory-II Scale, and the modified Depression Stigma Scale. A multiple-mediation analysis procedure was applied to analyze the data. Each indirect effect of self-stigma (B = −0.0974, bootLLCI, bootULCI: −0.1742, −0.0436) and depression (B = −0.0471, bootLLCI, bootULCI: −0.1014, −0.0060) is statistically significant in the relationship between public stigma and attitudes toward psychiatric help. The individualized intervention for enhancing positive attitude or motivation for seeking help at the personal level of the nurse and depression tests—including regular physical health check-ups—is necessary.

## 1. Introduction

Nursing is a stressful and demanding profession which, inevitably and subsequently leads to high levels of work-related stress and a high rate of turnover, worldwide [1]. The emergence of integrated nursing care service systems for dealing with new and complicated diseases have increased nurses’ work-related stress levels [2]. Previous studies have found that the intensity of the stressor (in exceeding an individual’s tolerance threshold) is linked to higher rates of depression [3]. Moreover, registered nurses suffer from depression at almost twice the rate of individuals working in other professions [3]. As nurses are the first point of contact most patients have in a clinic setting, and given that nurses comprise the highest percentage (68%) of health workers in Korea, their role is directly linked to the quality of medical service provided and received [4,5].

Among registered nurses, depression shows significant positive associations with aspects of job stress, burnout, intent to leave the profession, and somatic symptoms such as fatigue and trouble sleeping [6]. The greatest concern to the nursing profession is that depressed workers often exhibit low mood, have difficulty with concentration, and are accident prone. They are also significantly more limited in their ability to perform mental or interpersonal tasks, have worse time management skills, and have lower total work output than non-depressed workers. Thus, not only are hospital nurses with depression likely to suffer themselves, but their illness is also likely to impact their coworkers, and potentially the quality of care they provide [7]. As nurses provide health care services to patients for nearly 24 h a day, their mental health condition not only related to the quality of health care, but to patients’ safety. Saleh et al. [8] found that there is a highly significant positive correlation between depression and the frequency of medication errors. In addition, Garrouste-Orgeas et al. [9] found that symptoms of depression are an independent risk factor for medical errors. Therefore, preventing and managing depression among nurses is highly important—not only for their personal health, but for good quality healthcare service delivery.

The early detection and treatment of depression is affected by nurses’ attitude toward the condition and its management. Many individuals do not look for professional help for their psychiatric problems [10] and only consider asking for professional help after seeking non-professional help—such as by talking to immediate family, friends, and relatives [11]. Like other chronic diseases, early diagnosis and proper intervention are also emphasized in depression as it can prevent chronicity and reduce the pain caused by the disease [12]. However, among adults in Korea —including nurses—treating depression via professional psychiatric help is the lowest throughout the Organization for Economic Cooperation and Development (OECD) [13]. According to a survey regarding mental disorders in Korea (2016), mental health services usage by people with mood disorders, including depression, is 52.5%, while the rate of visits to psychiatrists is 40.4%, which is relatively low compared to more-developed countries [13]. A help-seeking attitude is a strong predictor of one’s attitude toward psychiatric help [11]. That is, if nurses’ attitude to psychiatric help is good, they would be more willing to accept psychiatric help. However, there are no previous studies reporting the “professional help-seeking” attitude and behavior of nurses. Therefore, it is necessary to study nurses’ attitudes and behaviors in regard to seeking help so as to predict their attitudes in seeking help for depression.

Stigma is one of the major barriers to seeking treatment for depression [14,15,16,17]. Schwenk et al. [18] also reported that stigma associated with depression, along with the use of mental health care services, could impede individuals from seeking treatment for the condition. The stigma related to mental health problems can be divided into two categories: public stigma—which is defined as the stereotypes, prejudices, and discriminations an individual believes are held by the general public—and self-stigma—which is defined as the internalization of public stigma, or an individual’s own stigmatizing beliefs, attitudes, and prejudices about those with mental disorders (including themselves) [19]. Self-stigma includes internalized public stigma and can be measured through the Internalized Stigma Mental Illness (ISMI) scale and the Self-Stigma Scale-Short (SSS-S) [20]. However, because self-stigma (defined as stigmatized individuals who accept and endorse the stereotype, prejudice, and discrimination on their characteristics), perceived stigma (defined as stigmatized individuals who are aware of the stereotype, prejudice, and discrimination on their characteristics), and experienced stigma (defined as stigmatized individuals who receive prejudice and discrimination from others) are different concepts, self-stigma needs careful investigation [21,22]. Therefore, it is necessary to consider the variations of public and self-stigma that may impede a nurse’s attitude toward getting psychiatric help. 

Decreasing the existing public stigma surrounding depression would be one potential facilitator in nurses seeking professional help for depression [23]. Public stigma would have an impact on self-stigma and, as such, will have an impact on help-seeking behavior [24]. However, there have been mixed results concerning the impact of public and self-stigma on individuals’ attitudes toward psychiatric help [23,25]. Furthermore, very few studies have been conducted on nurses; the only studies which can be found among the existing literature concern medical and nursing students [26]. Therefore, it is necessary to explore the order of influence of stigma on the attitude toward psychiatric help. The difference in approaches toward public and self-stigma will be helpful in educating nurses, and providing an intervention point for the lowering of both stigmas consecutively while seeking psychiatric help for depression at the right time. Interventions—such as education, consumer contact, cognitive behavior therapy, acceptance and commitment therapy, mindfulness, narrative enhancement, and others—have been mainly conducted so as to reduce self-stigma [27]. Likewise, public stigma can be further reduced through campaigns or continuous media exposure; however, it is necessary to know which stigma (self or public) further influence the attitude toward psychiatric help. Thus, nurses’ mental health—and especially depression—should be managed and treated at an early stage for the sake of patients’ health and safety, along with their own.

This study aimed to examine the mediating effects of self-stigma and depression on both public stigma and nurses’ attitude toward psychiatric help. The specific research purposes were as follows: First, the correlation between public stigma, nurses’ help-seeking behavior, self-stigma, and depression was identified. Second, whether depression and self-stigma are serial-mediated by public stigma and attitude toward psychiatric help was examined.

## 2. Materials and Methods

### 2.1. Sampling and Data Collection

This was a cross-sectional study. The participants of this study were recruited from one general hospital located in the southern part of South Korea. According to G*Power 3.1.9 program, a for multiple regression analysis using significance level 0.05, medium effect size 0.15, and power 95%, the minimum number of samples was 153 [28]. Since the number of participants needed for statistical significance is 5–10 times the parameters in path analysis, at least 100 participants were required. Based on this analysis, we distributed 200 surveys with 20% missing rate and 184 were collected (response rate = 92%) and used for analysis. Data were collected in the period between June and August 2018 using a self-administered survey. Before recruitment began, the study was approved by the University Institutional Review Board (IRB); the primary investigator (PI) also received permission from the general hospital. The consent forms and questionnaires were enveloped with a stamp and sent to nurses who agreed to participate in this study. The PI obtained written consent from all the participants.

### 2.2. Instruments

#### 2.2.1. Attitude Toward Psychiatric Help 

The Korean version of the 10-item “Attitudes toward psychiatric help” (ASPH) survey [29], which employs a 5-point Likert-type response scale, was used to measure the attitude toward seeking professional help for depression [30]. This scale measured one’s general tendency to seek mental healthcare services for any own mental health issue. Higher totals of scores indicated more positive attitudes toward seeking professional help. Higher total scores also indicate a greater level of positive attitudes toward seeking professional help. Items 2, 4, 8, 9, and 10 were reverse-scored as they sought input regarding a negative attitude; for example, Item 10 reads: “Personal and emotional troubles, like many things, tend to work out by themselves” [30]. At the time of development, the Cronbach’s alpha was 0.76 [30] and the current study’s alpha is 0.765. The Kaiser–Meyer–Olkin (KMO) value was found to be 0.792 and the Bartlett test exhibited significant results (x^2^ = 480.606, df = 45, *p* < 0.001). 

#### 2.2.2. Depression 

The Beck Depression Inventory-II (BDI-II), which consists of 21 items, was used to detect depression [31]. Each item is selected from four statements with 0–3 points, with the scores of each item summed and scored. The total score range is 0–63 points: 13 points or less indicate minimal depression; 14–19 points indicate mild depression; 20–28 points indicate moderate depression; and 29 points or more indicate severe depression [32]. Items dealt with depressive symptoms, including weight loss, change in body image, somatic symptoms, loss of energy, sleep loss, and appetite loss, as well as sadness and loss of interests [31]. The Korean version of BDI-II (K-BDI-II) was purchased from the Korean Psychology Association [33]. The Cronbach’s alpha for the BDI-II in population is 0.909. Furthermore, the KMO value is 0.868 and the Bartlett test is significant (x^2^ = 1209.002, df = 231, *p* < 0.001).

#### 2.2.3. Depression Stigma 

Depression stigma was measured by revising the tool designed by Griffiths and colleagues [34], and the modified Korean version of the depression stigma scale (DSS) was used [35]—the reliability of which was tested by Jeong et al. [35,36]. This tool consists of six self-stigma questions and nine public stigma questions. The responses were coded on a 4-point Likert scale, with the total score ranging from 0 to 60; higher scores indicate a greater level of stigma surrounding depression and its treatment. The Cronbach’s alpha for self-stigma is 0.655, 0.858 for public stigma, and 0.843 for total stigma. The KMO value is 0.779 and the Bartlett test was significant (x^2^ = 1066.549, df = 105, *p* < 0.001). 

### 2.3. Ethical Considerations

Before recruitment began, the study was approved by the University IRB (Approval No. KYU-2018-059-01). The written consent form—including a statement about voluntary participation and protection of anonymity and confidentiality—was obtained from all participants. 

### 2.4. Data Analysis

Correlation analysis was conducted—by applying Pearson’s correlation coefficient—so as to examine correlations among the attitudes toward psychiatric help, depression stigma, and depression. The correlation analysis was performed using SPSS version 25.0 (IBM Corp., Armonk, N.Y., USA) [37] and Process Macro version 3.4 [38]. The age and gender of the participants were included as covariate variables in the analysis. Full Information Maximum Likelihood (FIML) procedure, which is robust to non-normality and missing data, was applied. For testing the hypothesis of serial multiple mediation analysis, Process Macro model 6 and bootstrapping was conducted with a 95% confidence interval (CI) [39]. An indirect effect was considered to be significant if its 95% bootstrap CIs from 10,000 bootstrap samples did not include zero.

## 3. Results

### 3.1. Sample Characteristics

The average age of the study subjects is 26.56 years, while the average amount of experience amounts to 4.05 years. Among the study subjects, 174 (95%) participants are women; 161 (88%) participants are unmarried; and 164 (88%) participants are graduates. The participants of the study are distributed throughout different units within the hospital: 47 (26%) work in the intensive care unit; 44 (24%) work in the internal unit; 33 (18%) work in the surgical unit; 21 (11%) work in the operating room; 20 (11%) work in the emergency room; 13 (7%) work in other units; and 6 (3%) work in the nursing care integration unit (as shown in Table 1).

### 3.2. Correlations Among Variables

Table 2 Shows the correlation between the main variables. The attitude toward psychiatric help is significantly correlated with depression (r = −0.244, *p* < 0.01) and self-stigma (r = −0.238, p < 0.01), but is not significantly related to public stigma. Self-stigma showed significant correlation with attitudes toward psychiatric help (r = −0.238, *p* < 0.01) and public stigma (r = −0.404, *p* < 0.001). Depression showed a significant correlation with attitudes toward psychiatric help (r = −0.244, *p* < 0.01), but not with self-stigma and public stigma. 

### 3.3. Mediating Effects of Self-Stigma and Depression in The Relationship between Public Stigma and Attitudes Toward Psychiatric Help

The mediating effects of self-stigma and depression in the relationship between public stigma and attitudes toward psychiatric help are shown in Table 3 and Figure 1. Public stigma has a positive effect on self-stigma (β = −0.230, *p* < 0.001) and negatively affects attitudes toward psychiatric help (β = −0.423, *p* < 0.05). Public stigma positively affects depression (β = −0.278, *p* < 0.05) and depression has a negative influence on attitudes toward psychiatric help (β = −0.169, *p* < 0.05). In addition, public stigma has a positive effect on self-stigma (β = −0.230, *p* < 0.001), self-stigma has a negative effect on depression (β = −0.445, *p* < 0.01), and depression has a negative effect on attitudes toward psychiatric help (β = −0.169, *p* < 0.05). 

The direct and indirect effects of self-stigma and depression were examined; it was observed that the direct effect of public stigma and attitudes toward psychiatric help are not significant (direct effect = 0.0759, bootLLCI, bootULCI: −0.0581, 0.2100). The total size of the indirect effect is −1.288 (bootLLCI, bootULCI: −0.2187, −0.0578), and was found to be statistically significant as there are no zeroes between LLCI and ULCI in the confidence interval. As a result of simple mediation effect verification, X → M1 → Y is −0.0974 (bootLLCI, bootULCI: −0.1742, −0.0436) and X → M2 → Y is −0.0471 (bootLLCI, bootULCI: −0.1014, −0.0060), and each mediating effect is found to be significant. As a result of verifying the serial mediating effect, X → M1 → M2 → Y is−0.0174 (bootLLCI, bootULCI: −0.0002, −0.0428), which is not considered to be statistically significant. Through this, the serial mediation effects of self-stigma and depression are confirmed in the relationship between public stigma and attitudes toward psychiatric help.

## 4. Discussion 

The purpose of this study was to identify the serial mediation of self-stigma and depression in public stigma and depressed nurses’ help-seeking behavior.

First, attitudes toward psychiatric help is associated negatively with depression and self-stigma. The higher is the level of depression, the higher is the level of self-stigma, and the lower is the positive attitude toward psychiatric help. This result is consistent with that of an earlier study which reports that public stigma and self-stigma are independently related to attitudes toward seeking psychiatric help [14], and that self-stigma is negatively associated with help-seeking. A depressed mood is associated with delayed help-seeking and symptom recognition, even among those who have previously received treatment for depression [40]. Perceived public stigma and self-stigma are significantly related to each other, as well as to attitudes toward psychiatric help and a willingness to seek counseling [24]. In other words, people with higher levels of depression and high public and self-stigma have low professional treatment rates. However, in this study, public stigma and attitude toward psychiatric help are not related—but some studies do report the relationship between public stigma and professional psychotherapy [14,24]. Another study also shows that self-stigma is significantly and negatively associated with measures of help-seeking (a perceived need and use of psychotropic medication, therapy, and nonclinical sources of support), whereas public stigma is not significantly associated with help-seeking [41] and does not appear to have a significant impact on seeking psychiatric help [42]. This shows that there is a greater connection between the attitude toward psychiatric help and self-stigma as compared to public stigma. However, it is necessary to investigate this relationship more clearly through subsequent studies.

Secondly, it was found that self-stigma and depression are mediated by public stigma in influencing attitude toward psychiatric help. This is consistent with previous findings that public stigma is mediated by self-stigma in pathways that influenced the attitude or behavior of psychiatric help [23,24,25]. This means that, in addition to the existing literature that mainly claims public stigma in psychotherapy approaches, it is imperative to understand the self-stigma of nurses and how to lower it so as to improve their attitudes toward seeking psychiatric help and access to psychotherapy. Moreover, nurses are said to suffer from personal and professional difficulties due to depression, as they do not easily receive expert help on their psychiatric problems, usually only considering it last [10,11]. Therefore, at the level of hospitals and nursing personnel, it is necessary to detect depression early through regular depression tests and to improve the accessibility to psychiatric treatment by improving the work environment and overall institutional awareness. In addition, personalized education and interventions should be planned to identify characteristics of individual nurses and consider them through interviews and regular meetings within the organization.

As shown in this study, public stigma affects self-stigma. Therefore, self-stigma can be reduced by reducing public stigma toward depression through improved work welfare, such as campaigns of anti-stigma for depression, providing education on the detection and treatment of depression in the organization, and permitting nurses leave of absence and flexible working hours during the treatment for depression. According to the results of this study, and given that depression mediates the relationship between public stigma and attitude, it is necessary to include depression assessment in regular health checkups provided to employees for the means of its early detection, and to ensure that these results are not utilized in personnel scores and organizational life. This implication would be practical since the educational program for improving mental health literacy could enhance the knowledge about mental disorders, lower misbelief about mental disorders and their treatment, but could not enhance the actual seeking psychiatric help [43]. Therefore, it implies that nurses’ mental health issue including depression should be screened before or while applying educational program for enhancing mental health literacy in order to enhance practical effect on help-seeking behavior. Furthermore, the nursing department and nursing association need to prepare guidelines and recommendations for depression tests and education for nurses so as to ensure the safety of patients, as well as the health of nurses. These efforts by individual nurses and nursing organizations will improve the attitude toward psychiatric help and depression treatment rates.

With regard to depression in nurses, the attitude or motivation for seeking help at the personal level is important. This will reduce nurses’ depression by improving their attitude toward psychiatric help and accessibility of psychiatric help, thereby increasing their concentration on their work, further reducing the number of medical errors [7,8]. As such, to lower individual stigma and be treated early, the efforts of individual nurses—as well as the efforts of nursing departments, hospitals, and nursing associations—must be coordinated.

## 5. Recommendation for Future Research

Future research should address the following: firstly, other influencing factors identified in previous studies as variables related to depression—such as organizational seniority, job stress, stress coping styles, and body mass index—and actual behavior as well as attitude toward seeking help should be examined. Secondly, the effects of attitude toward psychiatric help and depression stigma between a depressed and non-depressed group should be identified. Thirdly, this study was conducted on nurses in hospitals; the study finding is, therefore, difficult to generalize to nurses in various fields. As such, through additional studies targeting professional personnel from various regions and medical institutions, a foundation should be prepared to facilitate the action of assisting nurses and medical professionals with depression working in local communities and medical institutions. Fourth, the participants of this study are young and have less clinical experience than expected. Participants may be confused with the findings of the study because adaptive abilities in new environments, along with interpersonal relationship skills, may still be immature. Lastly, all the instruments were self-reported—social desirability or recall bias may, thus, threaten the results. Therefore, we suggest a follow-up study that complements and addresses the above limitations.

## 6. Implications for Nursing Practice

It is extremely important to recognize the seriousness surrounding the low rate of seeking psychiatric help for mental health problems as a response to public and self-stigma. This is particularly important among nurses, as they are generally the first, and overall most important, individuals ensuring the safety of patients. As stigma is one of major barriers in seeking psychiatric help, it is important to lower both types of stigma related depression at the hospital level, since hospitals are the centers of workplace for nurses. Based on results from this study, individualized assessment and educational program for decreasing stigma related to depression and its treatment should be made, since self-stigma mediates the relationship between public stigma and attitudes toward psychiatric help. Furthermore, since depression mediates the relationship between public stigma and attitude towards psychiatric help, it is necessary to include depression assessment in regular health checkups provided to employees for the early detection thereof, and to ensure that these results are not utilized in personnel scores and organizational life. In addition, by providing self-help programs that can be used in various ways on and off-line, mental health can be improved. Nurses are required to increase the accessibility of the program because of irregular working hours and safety problems such as infections. Furthermore, governments and hospitals must create laws or regulations that regularly monitor the mental health of nurses as well as workers of psychiatric unit. This is an important part of protection for workers as much as physical damage that can occur in the working environment.

In summary, hospitals should plan educational programs for psychological interventions in nursing departments, and should further create an environment whereby a nursing association can actively implement these programs in a hospital setting. Additionally, nurses with severe stress, anxiety, and depression should be identified through consultation with mental health nurses and subsequently referred to external professional counseling centers or mental health clinics. Additionally, nurses with depression should be identified through consultation with mental health nurses and referred to external professional counseling centers or mental health clinics. In addition to depression, these interventions are also necessary in cases of mental illnesses such as PTSD, anxiety disorders, and obsessive-compulsive disorders.

## 7. Conclusions

The present study was the first to explore the mediating effects of self-stigma and depression in the relationship between public stigma and attitude toward psychiatric help among Korean nurses. Self-stigma and depression each had an indirect effect on the relationship between public stigma and attitudes towards psychiatric help. Interventions or programs are needed to lower self-stigma to promote nurses’ attitude to toward psychiatric help.

## Figures and Tables

**Figure 1:** A serial mediation analysis of personal stigma and depression on public stigma to attitudes toward psychiatric help.

**Table 1:** Characteristics of participants (N =184).

Characteristics	Categories	Mean (±SD) or n (%)
Age		26.56 (±3.59)
Total career year		4.05 (±3.94)
Gender	Male	10 (5%)
	Female	174 (95%)
Marital status	Single	161 (88%)
	Married	23 (13%)
Education	College	20 (12%)
	University	164 (88%)
Department		
	Internal unit	44( 24%)
	Surgical unit	33 (18%)
	emergency room	20 (11%)
	Intensive care unit	47 (26%)
	operating room	21 (11%)
	Nursing Care Integration	6 (3%)
	Other (Gynecology, Psychiatry)	13 (7%)

**Table 2:** Correlations among variables of nurses (N= 184).

	Help-Seeking	Depression	Self-Stigma	Public Stigma
Depression	−0.244 **			
Self-stigma	−0.238 **	−0.069		
Public stigma	−0.049	−0.121	−0.404 ***	−1
Mean	−26.30	−12.05	−14.32	−26.53
SD	−5.345	−8.312	−3.533	−6.295

Note: ** *p* < 0.05, *** *p* < 0.001. SD, Standard deviation.

**Table 3:** A Serial Mediation Analysis of Personal Stigma and Depression on Public Stigma to Attitude Toward Psychiatric Help.

	b	se	boot se	bootLLCI	bootULCI
direct	0.0759	0.0679		−0.0581	0.2100
indirect					
total	−0.1271		−0.0407	−0.2187	−0.0578
x → m1 → y	−0.0974		−0.0336	−0.01742	−0.0436
x → m2 → y	−0.0471		−0.0251	−0.01014	−0.0060
x → m1 → m2 → y	−0.0174		−0.0110	−0.0002	−0.0428

Note: Number of bootstrap samples for bias corrected bootstrap confidence intervals: 10,000. Level of confidence for all confidence intervals: 95%. x, public stigma; m1, self-stigma; m2, depression; y, attitude toward psychiatric help. LL, lower level; UL, upper level.
